The article "Fine-granularity inference and estimations to network traffic for SDN" was retracted in 2025. Reasons: unreliable results or conclusions; concerns about the peer review; concerns about the article.

# Fine-granularity inference and estimations to network traffic for SDN

**DOI:** 10.1371/journal.pone.0194302

**Published:** 2018-05-02

**Authors:** Dingde Jiang, Liuwei Huo, Ya Li

**Affiliations:** 1 School of Astronautics and Aeronautic, University of Electronic Science and Technology of China, Chengdu, China; 2 School of Computer Science and Engineering, Northeastern University, Shenyang, China; University College London, UNITED KINGDOM

## Abstract

An end-to-end network traffic matrix is significantly helpful for network management and for Software Defined Networks (SDN). However, the end-to-end network traffic matrix's inferences and estimations are a challenging problem. Moreover, attaining the traffic matrix in high-speed networks for SDN is a prohibitive challenge. This paper investigates how to estimate and recover the end-to-end network traffic matrix in fine time granularity from the sampled traffic traces, which is a hard inverse problem. Different from previous methods, the fractal interpolation is used to reconstruct the finer-granularity network traffic. Then, the cubic spline interpolation method is used to obtain the smooth reconstruction values. To attain an accurate the end-to-end network traffic in fine time granularity, we perform a weighted-geometric-average process for two interpolation results that are obtained. The simulation results show that our approaches are feasible and effective.

## Introduction

With extensive applications of new generational information technologies, smart city, Internet of Things and Software Defined Networks (SDN) applications have explosively grown. High-speed backbone networks for supporting these applications carry huge network traffic loads. The backbone network scale has been expanding, and its speed has continuously improved [1–2]. These changes have brought great challenges to network measurement techniques. To measure the performance of networks, network operators need to collect traffic data from a large number of network test nodes [2–3]. However, only an OC48 link can collect hourly traffic up to 600 GB. We must spend a lot of resources to store, transfer and handle the traffic data, since incorrect methods can cease network measurements. Therefore, in next-generation networks such as SDN, large-scale and high-speed sampling techniques have become one of main choices to measure and monitor communications networks [3–5]. These techniques significantly reduce the amount of measuring data and can also avoid adding the extra overhead brought by network measurements. However, sampling techniques can only obtain incomplete measured data that affect the correct analysis of network monitoring, network management, and performance assessment [4–8]. This may lead to an incorrect final decision. Hence, how to accurately derive the end-to-end traffic in finer time granularity from the limited sampling information has aroused extensive academic attention in recent years.

The article "Fine-granularity inference and estimations to network traffic for SDN" was retracted in 2025. Reasons: unreliable results or conclusions; concerns about the peer review; concerns about the article.

End-to-end traffic estimation has received extensive research attention and now has become the most important research topic of the IP network [9–11]. Cao et al. [12] used the expectation-maximization algorithm to estimate the origin-to-destination (or end-to-end) flow. Xie et al. [13] introduced a fast low-rank matrix method to detect network traffic anomalies. Zhang et al. [14] studied end-to-end traffic inference in a large-scale IP backbone network. Moreover, they also investigated the end-to-end network traffic in point-to-point and point-to-multipoint cases [15]. Juva et al. studied the sensitivity of the existing end-to-end network traffic recovery approaches [16]. Additionally, Fumo et al. used a joint spatial and temporal approach to classify mobile traffic demands [17]. Stoev et al. found that the probability model that combined traditional single-link (single-flow) traffic models with routing could capture the global behavior of network traffic [18]. Some synthetic methods have been presented to generate end-to-end network traffic in order to conduct normal network activities [2]. Spatio-temporal compressive sensing sufficiently considers sparsity in the end-to-end network traffic [1]. Current studies have found that network traffic has long-range dependence and a self-similar nature [19–22]. In other words, when the network traffic is measured at different time scales (milliseconds to hours), we find that network traffic has similar characteristics. Different these methods, SDN provides direct network flow measurements with a chance.

Our motivations include several aspects. Firstly, an accurate end-to-end network traffic matrix is very important and helpful for performing effective network managements and traffic engineering. Unfortunately, the direct measurements of them in the traditional network is prohibitive. Moreover, the end-to-end network traffic matrix's inferences and estimations are a huge challenge, and these methods have the larger estimation errors. Secondly, in contrast to traditional networks, SDN can provide better solutions to traffic measurements of network flows, which allows to directly obtain the end-to-end traffic via reading the flow counter in the OpenFlow switch. Compared with the estimation methods based on the Simple Network Management Protocol (SNMP) link load measurements, this can improve the traffic measurement accuracy. However, under the SDN framework, to obtain the measurement results in fine time granularity is still complex, difficult and prohibitive, particularly for the high-speed network. Thereby, based on SDN idea, it is necessary to construct a light-weight accurate method to obtain network traffic for network managements and designs. Thirdly, the sampling measurements for the end-to-end flow traffic can obtain their accurate sample value by the little measurement overhead, but the sampling results are too coarse for some applications (such as billing, real time traffic scheduling, traffic anomaly detection, and so forth). Fortunately, the matrix complement can obtain the finer-granularity traffic value based on the end-to-end sampling. Therefore, in this paper, underlying the SDN idea and framework, we consider how to construct a fine-granularity inference and estimations to the end-to-end network traffic from the sampling results in coarse time granularity.

The article "Fine-granularity inference and estimations to network traffic for SDN" was retracted in 2025. Reasons: unreliable results or conclusions; concerns about the peer review; concerns about the article.

Our main contributions in this paper are summarized as follows:

- We propose a new approach to attain the fine-granularity end-to-end network traffic for SDN. Extracting the accurate end-to-end network traffic matrix has far-reaching impacts on network planning, network optimization, and network dimensioning in SDN applications. However, with the successful application of new network technologies, network traffic has exponentially boomed. Attaining the needed traffic volume of flows in high-speed networks is a prohibitive challenge. We also perform the detailed theoretical derivation for the end-to-end reconstruction and estimation. Our method can effectively overcome these problems.
- We propose a system model of the end-to-end traffic recovery to attain the fine-granularity accurate traffic estimation from the coarse-granularity sampled traffic data. The sampling measurement is one possible choice for the ligh-weight end-to-end traffic measurement. We investigate how to recover the end-to-end network traffic in the fine time granularity from sampled traffic traces, based on the proposed model in this paper.
- We present several algorithms to implement our reconstruction method of the end-to-end traffic. Due to the fractal and self-similar features of network traffic, we employ the fractal interpolation method to reconstruct network traffic in finer time granularity. After doing so, we obtain one result that meets the fractal properties. Generally, although such a result can accurately capture the fractal and self-similar nature of network traffic, it is inconsistent with real network traffic due to the non-smoothing nature of fractal interpolation results. Accordingly, the cubic spline interpolation method is used to obtain the smooth reconstruction values. To attain the accurate network traffic in fine time granularity, we perform the weighted geometric average process for the two obtained interpolation results. In such a case, we can recover the network traffic in the needed time granularity.
- A larger amount of simulation experiments are conducted to validate our approach. We analyze in detail the reconstruction results in the different sampling granularities. The spatial and temporal estimation errors are carefully discussed and analyzed. Simulation results show that our approach is feasible and effective.

The article "Fine-granularity inference and estimations to network traffic for SDN" was retracted in 2025. Reasons: unreliable results or conclusions; concerns about the peer review; concerns about the article.

The rest of this paper is organized as follows. Section 2 introduces the system model of the end-to-end network traffic reconstruction. Section 3 describes our end-to-end network traffic reconstruction methods. Section 4 presents the simulation results and analysis. It evaluates the reconstruction errors, the impact of the sampling time granularity on performance, and the average performance improvement. Finally, we conclude our work in Section 5.

## System model

End-to-end traffic in a network reflects the volume of flows from the origin to the destination. All end-to-end traffic describes their flows in the given network. This gives us the network-wide traffic information, which is very important for traffic engineering and network design. As mentioned in [1,13,23–24], all end-to-end traffic traverses the network according to the routing configuration. Simultaneously, the end-to-end traffic flows on the same link and aggregates into linked traffic. Thus, end-to-end traffic, linked traffic, and the routing configuration information meet a linear constraint. For time *t*, the following equation is obtained:

z(t)=By(t) (1)

where *z*(*t*) = (*z*_1_(*t*),*z*_2_(*t*),…,*z*_*v*_(*t*))^*T*^ denotes all linked traffic. *z*_*i*_(*t*) represents the traffic amount of link *i* where *i* = 1,2,…,*v*. *T* is the matrix transpose operator. *v* represents the total number of links in a given network. *y*(*t*) = (*y*_1_(*t*),*y*_2_(*t*),…,*y*_*u*_(*t*))^*T*^ is all end-to-end network traffic in a given network (namely, traffic matrix). *u* is the total number of origin-destination node pairs. *y*_*j*_(*t*) is the traffic amount of origin-destination flow *j*. *B* = (*b*_*ji*_)_*u×v*_ represents the routing matrix that describes the routing configuration information in the given network. *b*_*ji*_ = 1 if the origin-destination flows from *j* through the link *i*, and *r*_*ij*_ = 0 otherwise. Generally, *B* is obtained by network topology and routing configuration information.

In contrast to linked traffic *z*(*t*), end-to-end traffic *y*(*t*) is more significant for network management and network operations. As shown in Eq (1), end-to-end traffic is hidden in linked traffic. The inference method is primarily used to obtain the end-to-end traffic. Although some such approaches can obtain considerably accurate values for the end-to-end traffic, reconstruction errors always exist due to indirect measurements. In this paper, we perform the direct measurement to quickly obtain the end-to-end traffic in the coarser time granularity. Fig 1 denotes a certain direct measurement case of end-to-end traffic in coarse time granularity. From Fig 1, we can clearly see that the sampling measurement has loss, which cannot reflect the real end-to-end traffic in the given network. Therefore, an approach to accurately recover and reconstruct the end-to-end traffic is significantly important.

The article "Fine-granularity inference and estimations to network traffic for SDN" was retracted in 2025. Reasons: unreliable results or conclusions; concerns about the peer review; concerns about the article.

**Fig 1:** Direct measurement of the end-to-end traffic in coarse time granularity.

For SDN applications, network traffic has an important impact on the controller decisions [25–26]. Therefore, traffic recovery is important for network activities [27–28]. Fig 2 describes the system model of the end-to-end traffic recovery from coarse time granularity to fine. In this model, we use inverse sampling technologies to attain the accurate end-to-end traffic in fine time granularity. Without loss of generality, we assume that when the sampling interval is 5 × *m* minutes, where *m* > 1, the sampling value of end-to-end traffic is *y*_*m*_(*t*). We use the interpolation method to achieve the inverse sampling process, which can utilize the sampling values to reconstruct the fine-time-granularity traffic. ${\hat{y}}_{f}(t)$ represents the origin-destination traffic reconstructed by the fractal interpolation method such that $y_{m}(t)\Rightarrow {\hat{y}}_{f}(t)$. ${\hat{y}}_{s}(t)$ represents the end-to-end traffic reconstructed by the cubic spline interpolation method such that $y_{m}(t)\Rightarrow {\hat{y}}_{s}(t)$. Then, we make full use of the constraint relationship denoted in Eq (1) to attain the recovered end-to-end traffic ${\hat{y}}_{fp}(t)$ and ${\hat{y}}_{sp}(t)$, which correspond to ${\hat{y}}_{f}(t)$ and ${\hat{y}}_{s}(t)$, respectively. Moreover, according to ${\hat{y}}_{fp}(t)$ and ${\hat{y}}_{sp}(t)$, we employ the weighted geometric average to the needed end-to-end traffic $\hat{y}(t)$. Thus,

$$\hat{y}(t)={\left({\hat{y}}_{fp}(t)\right)}^{b_{1}}{\left({\hat{y}}_{sp}(t)\right)}^{\left(1-b_{1}\right)}$$ (2)

where *b*_1_ represents the weighted coefficient, and 0 ≤ *b*_1_ ≤ 1. Eq (2) combines the advantages of the fractal interpolation and the cubic spline interpolation methods to attain the accurate reconstruction result $\hat{y}(t)$. The fractal interpolation result ${\hat{y}}_{fp}(t)$ can effectively characterize the self-similar nature of network traffic, while the cubic spline interpolation estimation ${\hat{y}}_{sp}(t)$ can capture its highly dynamic change. This guarantees that $\hat{y}(t)$ can generate the optimal reconstruction traffic.

The article "Fine-granularity inference and estimations to network traffic for SDN" was retracted in 2025. Reasons: unreliable results or conclusions; concerns about the peer review; concerns about the article.

**Fig 2:** System model of the end-to-end traffic recovery.

## End-to-end traffic estimation

This section discusses our algorithm, which is based on fractal interpolation, cubic spline interpolation and the weighted geometric average algorithm, according to the system model shown in Fig 2.

### Fractal interpolation reconstruction

Fractal theory can describe the regularity of many irregular things and phenomena in the world. At present, it has a wide range of applications in natural, economic and social sciences [19]. One of the most important properties of fractal theory is that it must have a self-similarity. Self-similarity refers to the similarity existing between the whole and part of the system or between two separate parts. Current studies show that network traffic holds an obvious long-range dependent and self-similar nature. Furthermore, researchers have found that the packet lengths of TCP, FTP, video and other data have self-similarity that do not meet the exponential distribution. Moreover, they also discovered that the packet length distribution was a step function, and the length of the flow followed a log-normal distribution [20–21].

From the view of network topology, the current topology between the entire network and the segment network has the characteristics of self-similarity. From the view of the data contents from networks, network traffic is self-correlated. The distribution of the network files (including the file that the user requested, the file that was actually transferred, the time of file transfer, and the file’s storage in the server-side) is a heavy-tailed distribution. Furthermore, from the transfer process of the network traffic point of view (including the application layer, the network transportation layer and the physical link layer), the self-similarity nature can be observed. The application layer is the data source of network communications [20]. It displays the self-similarity properties within a wide range of time, which is reflected in the distribution of its file size and the distribution of free time.

By analyzing the message size that comes from the traffic of the world wide web server, researchers have found that the distribution of the document obeys the heavy-tailed distribution [21]. Furthermore, through the analysis of Telnet and FTP, researchers have also found that the burst degree and the data size are also in line with the heavy-tailed distribution. The transportation layer of networks contains a series of protocols, such as the use of flow control and congestion control, to implement the upper-layer services of network communication. Both network retransmission and congestion control mechanisms become the factors that induce self-similarity. The transportation layers of networks realize transmissions and are dependent on the availability of network resources [21]. These resource include the buffering capacity and network bandwidth. The buffer can temporarily accommodate multiple network traffic. Its size directly affects the loss rate of packets and queuing delay. Network bandwidth determines the throughput of networks and decides the pros and cons of network performance. The self-similarity of network protocols in the higher level can be mapped to its underlying layer. For example, we can map the heavy-tailed characteristics of the file distribution in the application layer to the network layer so that it also has self-similarity. Likewise, this feature of the network layer will also be mapped to the data-link layer and make the network traffic have self-similarity. For the end-to-end traffic of big-time granularity, we can take advantage of its characteristics of fractal and self-similarity and then reconstruct it using fractal interpolation theory. In general, if we use fractal interpolation, we need to obtain an accurate function of fractal interpolation.

The article "Fine-granularity inference and estimations to network traffic for SDN" was retracted in 2025. Reasons: unreliable results or conclusions; concerns about the peer review; concerns about the article.

According to the above discussion and our system model in Fig 2, for the measurement value *y*_*g*_(*t*) of end-to-end network traffic in the certain time granularity *g* and the given measurement duration [0,*z*], we create the following set of points:

$$\{(t,y_{g}(t))|t\in [0,z],y_{g}(t)\in R\},$$ (3)

where *R* denotes the real number domain.

For the sampling measurement process, time *t* is discretized. Then, Eq (3) can be converted as follows:

$$\{(n_{s},y_{g}[n_{s}])|n_{s}\in Z,y_{g}[n_{s}]\in R\},$$ (4)

where *n*_*s*_∈{0,1,…,*N*} denotes the sampling time slots and *n*_*s*_∈*Z*, *N* is the total time slots of the sampling measurement, and where *R* denote the real number domain.

According to Eq (4) and the fractal interpolation function theory, we can easily create the below interpolation function series:

$$\{f_{n_{s}}(.)|y_{g}[n_{s}]=f_{n_{s}}(n_{s}),n_{s}\in \{0,1,\ldots ,N\}\}.$$ (5)

For *y*_*g*_[*n*] = [*y*_*g*_[0],…,*y*_*g*_[*N*]] and *n* ∈ {1,2,…,*N*}, the fractal interpolation function can be denoted as:

$$f(.)=\{f_{0}(.),f_{1}(.),\ldots ,f_{N}(.)\}.$$ (6)

In Eq (6), *f*_*i*_(.) (where *i*∈{1,2,…,*N*}) denotes the fractal interpolation function at point *i*, while *f*(.) the fractal interpolation function at all the points. Furthermore, the following equation holds:

$$f_{k}\left(\begin{array}{c} n\\ y_{g}[n] \end{array}\right)=\left(\begin{array}{cc} \alpha_{k} & 0\\ \beta_{k} & \gamma_{k} \end{array}\right)\left(\begin{array}{c} n\\ y_{g}[n] \end{array}\right)+\left(\begin{array}{c} \varepsilon_{k}\\ \delta_{k} \end{array}\right)$$ (7)

where *k*∈{1,2,…,*N*}. For endpoints (0,*y*_*g*_[0]) and (*N*,*y*_*g*_[*N*]), the fractal interpolation function *f*(.) is satisfied with the following two equations:

$$\left\{ \begin{array}{l} f_{k}\left(\begin{array}{c} 0\\ y_{g}[0] \end{array}\right)=\left(\begin{array}{c} k-1\\ y_{g}[k-1] \end{array}\right)\\ f_{k}\left(\begin{array}{c} N\\ y_{g}[N] \end{array}\right)=\left(\begin{array}{c} k\\ y_{g}[k] \end{array}\right) \end{array}\right.$$ (8)

where *k* ∈ {1,2,…,*N*}.

The article "Fine-granularity inference and estimations to network traffic for SDN" was retracted in 2025. Reasons: unreliable results or conclusions; concerns about the peer review; concerns about the article.

According to the fractal interpolation function theory and Eqs (7) and (8), we let *γ*_*k*_∈(−1,1). Then, the affine transformation coefficient can be obtained:

$$\left\{ \begin{array}{l} \alpha_{k}=1/N\\ \varepsilon_{k}=N(k-1)/N\\ \beta_{k}=(y_{g}[k]‑y_{g}[k-1])/N‑\gamma_{k}(y_{g}[N]‑y_{g}[0])/N\\ \delta_{k}=Ny_{g}[k-1]/N‑\gamma_{k}y_{g}[0] \end{array}\right.$$ (9)

In terms of the above discussion and Eqs (4)–(9), given the sampling measurement value *y*_*g*_(*n*) with the coarse time granularity, we can easily reconstruct the end-to-end traffic ${\hat{y}}_{g}(k)$ with the fine time granularity using the fractal interpolation function theory. Without the loss of generality, suppose our reconstruction granularity is *v* time units. When the sampling interval is *v* × *j* (where *j*>1 and *j* ∈ *Z*) time units, the sampled network traffic is *y*_*v*,*j*_. If the data acquisition lasts *t*(0<*t*<*v*×*j*×*N*) time units, then each end-to-end flow has a total of *N* sampled data. Reconstructing the end-to-end traffic of *v* time units requires (*j*−1)×*N* interpolation points. The sampling points are *u*_*v*,*j*,*k*_ (*k* = 1,2,…,*N*) and *u*_*v*,*j*_ = (*u*_1_,*u*_2_,…*u*_*N*_). Using Eqs (4)–(9), the following equation can be obtained:

$$\left(\begin{array}{c} {\hat{n}}_{f,v,j}^{k}\\ {\hat{y}}_{f,v,j}^{k} \end{array}\right)=f_{k}\left(\begin{array}{c} u_{v,j}\\ y_{v,j} \end{array}\right)=\left(\begin{array}{c} \alpha_{k}\;0\\ \beta_{k}\;\gamma_{k} \end{array}\right)\left(\begin{array}{c} u_{v,j}\\ y_{v,j} \end{array}\right)+\left(\begin{array}{c} \varepsilon_{k}\\ \delta_{k} \end{array}\right)$$ (10)

where ${\hat{n}}_{f,v,j}^{k}$ and ${\hat{y}}_{f,v,j}^{k}$ respectively denote the time slots and the fractal interpolation results corresponding to the sampling network traffic *y*_*v*,*j*_ and the time granularity *v* after performing the fractal interpolation. Furthermore, *k*∈{1,2,…,*N*}.

The article "Fine-granularity inference and estimations to network traffic for SDN" was retracted in 2025. Reasons: unreliable results or conclusions; concerns about the peer review; concerns about the article.

Then, the reconstruction results $\left({\hat{n}}_{f}^{},{\hat{y}}_{f}^{}\right)$ using the fractal interpolation method are as follows:

$$\left\{ \begin{array}{l} {\hat{y}}_{f}^{}=({\hat{y}}_{f,v,j}^{1},{\hat{y}}_{f,v,j}^{2},\ldots ,{\hat{y}}_{f,v,j}^{N})\\ {\hat{n}}_{f}^{}=({\hat{n}}_{f,v,j}^{1},{\hat{n}}_{f,v,j}^{2},\ldots ,{\hat{n}}_{f,v,j}^{N}) \end{array}\right.$$ (11)

where ${\hat{n}}_{f}^{}$ and ${\hat{y}}_{f}^{}$ respectively denote the time slots and the fractal interpolation results corresponding to ${\hat{n}}_{f}^{}$.

The following states the detailed steps of our proposed fractal interpolation reconstruction approach.

**Algorithm 1:**

**Step1.** Give the sampling value *y*_*g*_(*t*) of the end-to-end network traffic.

**Step2.** According to Eqs (8) and (9), determine the parameters *α*_*k*_, *β*_*k*,_ *γ*_*k*,_ *ε*_*k*,_ and *δ*_*k*_.

**Step3.** According to Eqs (6) and (7), attain the fractal interpolation function *f*(.).

**Step4.** For each fractal interpolation function *f*_*k*_(.) where *k* = 1,2,…,*N*, perform the operation shown in Eq (10) and obtain the corresponding reconstruction result ${\hat{y}}_{f,v,j}^{k}$ of the end-to-end network traffic.

**Step5.** By Eq (11), obtain the fractal interpolation results ${\hat{y}}_{f}^{}$ and the corresponding time slots ${\hat{n}}_{f}^{}$.

### Cubic spline interpolation reconstruction

Although the fractal interpolation is able to obtain the reconstructed results of the end-to-end network traffic, its reconstruction error is relatively large, and the interpolation curve is not smooth. In this section, we discuss how to use the cubic spline interpolation to reconstruct the end-to-end traffic. Interpolation is one of the important methods of numerical approximation, which is based on the given values of the independent variable and approximate an unknown function. The cubic spline interpolation method can use a smooth curve to fit each trunk point. It constructs polynomials to form a smooth curve connecting all trunk points. Moreover, it can reconstruct the unique new sequence as long as it is given the original sample data and the reconstruction interval. We apply the cubic spline interpolation method to reconstruct the end-to-end network traffic.

According to the spline interpolation theory, to achieve network traffic with finer time granularity, we divide the sample interval of network traffic into *q* equal parts and then (on each subinterval) use the cubic Hermite interpolation method to deduce the cubic interpolation function *s*(*t*). Without the loss of generality, for the *kth* sample interval of network traffic [*k*,*k*+1], to interpolate the *q*−1 points of network traffic, assume that the following equation holds:

$$k=t_{0}^{k}<t_{1}^{k}<\ldots <t_{q-1}^{k}<t_{q}^{k}=k+1$$ (12)

Then, the cubic interpolation function *s*^*k*^(*t*) that corresponds to the interval [*k*,*k*+1] is satisfied with the following equation:

$$s^{k}(t_{i}^{k})=y_{g}^{i}[k],\;i=0,1,\ldots ,q$$ (13)

where $y_{g}^{i}[k]$ denotes the functional values corresponding to the time point $t_{i}^{k}$. *s*^*k*^(*t*) is no more than the cubic polynomial in each of the subintervals $\left[t_{i}^{k},t_{i+1}^{k}\right]$. Moreover, *s*^*k*^(*t*), (*s*^*k*^(*t*))', and (*s*^*k*^(*t*))" are all continuous in the range of [*k*,*k*+1].

The article "Fine-granularity inference and estimations to network traffic for SDN" was retracted in 2025. Reasons: unreliable results or conclusions; concerns about the peer review; concerns about the article.

Then, for the *kth* sample interval of network traffic [*k*,*k*+1], the cubic interpolation function *s*^*k*^(*t*) can be denoted as the following equation:

$$s^{k}(t)=a_{i}^{k}\frac{{\left(t_{i+1}^{k}-t\right)}^{3}}{6h_{i}^{k}}+a_{i+1}^{k}\frac{{\left(t-t_{i}^{k}\right)}^{3}}{6h_{i}^{k}}+(\frac{y_{g}^{i}[k]}{h_{i}}-\frac{a_{i}^{k}h_{i}}{6})(t_{i+1}^{k}-t)+(\frac{y_{g}^{i+1}[k]}{h_{i}^{k}}-\frac{a_{i+1}^{k}h_{i}^{k}}{6})(t-t_{i}^{k})$$ (14)

where $t\in [t_{i}^{k},t_{i+1}^{k}]$, *i* = 0,1,…,*q*, $h_{i}^{k}=t_{i+1}^{k}-t_{i}^{k}$, and $a_{i}^{k}$ $a_{i+1}^{k}$ are two parameters to solve.

The function *s*^*k*^(*t*) has a continuous second derivative at the sample points $t_{i}^{k}$. According to the cubic natural spline interpolation method, the following holds:

$$\left\{ \begin{array}{c} s^{k}(t_{i}^{k})=y_{g}^{i}[k]\\ (s^{k}(t_{0}^{k}))"=(y_{g}^{0}[k])"=0\\ (s^{k}(t_{q}^{k}))"=(y_{g}^{q}[k])"=0 \end{array}\right.$$ (15)

where *i* = 0,1,…,*q*. According to Eqs (14) and (15), we can solve parameters $a_{i}^{k}$ and $a_{i+1}^{k}$. Then, *s*^*k*^(*t*) is built.

Similar to subsection B, we assume that our reconstruction granularity is *v* time units. When the sampling interval is *v*×*j* (where *j*>1 and *j*∈*Z*) time units, the sampled network traffic is *y*_*v*,*j*_. If the data acquisition lasts *t* (0<*t*<*v*×*j*×*N*) time units, then each end-to-end flow has a total of *N* sampling data. Reconstructing the end-to-end traffic of *v* time units requires (*j*−1)×*N* interpolation points. The sampling points are *u*_*v*,*j*,*k*_ (*k* = 1,2,…,*N*) and *u*_*v*,*j*_ = (*u*_1_,*u*_2_,…*u*_*N*_). Using Eqs (12)–(15), the following equation can be obtained:

$$\left\{ \begin{array}{l} {\hat{y}}_{c,v,j}^{k}=s^{k}(t)\\ {\hat{n}}_{c,v,j}^{k}=u_{v,j,k} \end{array}\right.$$ (16)

where ${\hat{n}}_{c,v,j}^{k}$ and ${\hat{y}}_{c,v,j}^{k}$ respectively denote the time slots and the cubic interpolation results corresponding to the sampling network traffic *y*_*v*,*j*_ and time granularity *v* after performing the cubic interpolation. Furthermore, $t\in [t_{i}^{k},t_{i+1}^{k}]$, *i* = 0,1,…,*j*, and *k*∈{1,2,…,*N*}.

The article "Fine-granularity inference and estimations to network traffic for SDN" was retracted in 2025. Reasons: unreliable results or conclusions; concerns about the peer review; concerns about the article.

Then, the reconstruction results $\left({\hat{n}}_{c}^{},{\hat{y}}_{c}^{}\right)$ using the fractal interpolation method are as follows:

$$\left\{ \begin{array}{l} {\hat{y}}_{c}^{}=({\hat{y}}_{c,v,j}^{1},{\hat{y}}_{c,v,j}^{2},\ldots ,{\hat{y}}_{c,v,j}^{N})\\ {\hat{n}}_{c}^{}=({\hat{n}}_{c,v,j}^{1},{\hat{n}}_{c,v,j}^{2},\ldots ,{\hat{n}}_{c,v,j}^{N}) \end{array}\right.$$ (17)

where ${\hat{n}}_{c}^{}$ and ${\hat{y}}_{c}^{}$ respectively denote the time slots and the fractal interpolation results corresponding to ${\hat{n}}_{c}^{}$.

The following states the detailed steps about our proposed fractal interpolation reconstruction approach.

**Algorithm 2:**

**Step1.** Give the sampling value *y*_*g*_(*t*) of the end-to-end network traffic.

**Step2.** According to Eq (12), determine *q* equal intervals of network traffic.

**Step3.** According to Eqs (13)–(15), select the parameters $a_{i}^{k}$ and $a_{i+1}^{k}$.

**Step4.** Using Eq (14), determine the cubic interpolation function *s*^*k*^(*t*) corresponding to the interval [*k*,*k*+1], where *k* = 1,2,…,*N*.

**Step5.** Perform the operation shown in Eq (16) and obtain the corresponding reconstruction result ${\hat{y}}_{c,v,j}^{k}$ of the end-to-end network traffic.

**Step6.** Using Eq (17), obtain the fractal interpolation results ${\hat{y}}_{c}^{}$ and the corresponding time slots ${\hat{n}}_{c}^{}$.

### Weighted geometric average

Although the fractal and cubic spline interpolation methods can reconstruct the end-to-end network traffic, the reconstruction errors are inevitable. To further improve the reconstruction accuracy, we employ the weighted geometric average method to combine both interpolation approaches. We minimize the sum of squares of logarithm errors of the combination model to determine the optimal weighted coefficients.

According to the above discussion, for the reconstruction results ${\hat{y}}_{f}^{}$ and ${\hat{y}}_{c}^{}$ of the fractal and cubic spline interpolation methods, without the loss of generality, we assume that the following holds:

$$\left\{ \begin{array}{l} {\hat{y}}_{f}^{}=({\hat{y}}_{f}^{}(1),{\hat{y}}_{f}^{}(2),\ldots ,{\hat{y}}_{f}^{}(j\times N))\\ {\hat{y}}_{c}^{}=({\hat{y}}_{c}^{}(1),{\hat{y}}_{c}^{}(2),\ldots ,{\hat{y}}_{c}^{}(j\times N)) \end{array}\right.$$ (18)

Then, the weighted geometric average model for them can be denoted as:

$$\hat{y}(t)={\hat{y}}_{f}^{b}(t){\hat{y}}_{c}^{1-b}(t)$$ (19)

where *b* represents the weighted coefficient and 0≤*b*≤1. $\hat{y}(t)$ denotes the reconstruction results of the end-to-end network traffic at time *t* after performing the weighted geometric average. 0≤*t*≤*j*×*N* and *t*∈*N*. Eq (18) denotes the reconstruction results ${\hat{y}}_{f}^{}$ and ${\hat{y}}_{c}^{}$ via the fractal and cubic spline interpolation methods, respectively. Eq (19) obtain the reconstruction and estimation results according to our system model shown in Eq (2).

The article "Fine-granularity inference and estimations to network traffic for SDN" was retracted in 2025. Reasons: unreliable results or conclusions; concerns about the peer review; concerns about the article.

To calculate the weighted coefficient *b*, we assume *y*(*t*) represents the sample values of the end-to-end network traffic where 0≤*t*≤*j*×*N*. Using Eq (19), we obtain the following objective function:

$$\begin{array}{l} {E(t)}^{2}={\left(\ln\hat{y}(t)-\ln y(t)\right)}^{2}\\ \;={\left[b\ln\hat{y}(t)+(1-b)\ln{\hat{y}}_{c}(t)-\ln y(t)\right]}^{2}\\ \;={\left[b(\ln{\hat{y}}_{f}(t)-\ln y(t))+(1-b)(\ln{\hat{y}}_{c}(t)-\ln y(t))\right]}^{2}\\ \;=B^{T}D(t)B \end{array}$$ (20)

where 0≤*t*≤*j*×*N*. *D*(*t*) meets the following equation:

$$\begin{array}{c} D(t)={\left[\ln{\hat{y}}_{f}^{}(t)-\ln y(t),\ln{\hat{y}}_{c}^{}(t)-\ln y(t)\right]}^{T}\\ \left[\ln{\hat{y}}_{f}^{}(t)-\ln y(t),\ln{\hat{y}}_{c}^{}(t)-\ln y(t)\right] \end{array}$$ (21)

According to Eqs (20) and (21), for 0≤*t*≤*j*×*N*, we obtain the following objective function:

$$min\;E^{2}=\sum_{t=0}^{j\times N}E{\left(t\right)}^{2}=B^{T}\left(\sum_{t=0}^{j\times N}D(t)\right)B=B^{T}DB$$ (22)

Generally, *D* is a symmetric positive definite matrix. Therefore, for *B* = (*b*,1−*b*)^*T*^, *E*^2^>0. Then, Eq (22) can be converted into:

$$\left\{ \begin{array}{c} min\;B^{T}DB\\ s.t.\;b>0 \end{array}\right.$$ (23)

By solving Eq (23), we can the optimal weighted coefficient as follows:

$$b=\frac{\sum_{t=0}^{j\times N}E_{c}{\left(t\right)}^{2}-\sum_{t=0}^{j\times N}E_{f}(t)E_{c}(t)}{\sum_{t=0}^{j\times N}E_{f}{\left(t\right)}^{2}+\sum_{t=0}^{j\times N}E_{c}{\left(t\right)}^{2}-2\sum_{t=0}^{j\times N}E_{f}(t)E_{c}(t)}$$ (24)

The following equation holds:

$$1-b=\frac{\sum_{t=0}^{j\times N}E_{f}{\left(t\right)}^{2}-\sum_{t=0}^{j\times N}E_{f}(t)E_{c}(t)}{\sum_{t=0}^{j\times N}E_{f}{\left(t\right)}^{2}+\sum_{t=0}^{j\times N}E_{c}{\left(t\right)}^{2}-2\sum_{t=0}^{j\times N}E_{f}(t)E_{c}(t)}$$ (25)

where *E*_*f*_(*t*) and *E*_*c*_(*t*) are satisfied with:

$$\left\{ \begin{array}{c} E_{f}(t)=\ln{\hat{y}}_{f}^{}(t)-\ln y(t)\\ E_{c}(t)=\ln{\hat{y}}_{c}^{}(t)-\ln y(t) \end{array}\right.$$ (26)

According to Eqs (19)–(26), we can obtain the accurate reconstruction results $\hat{y}(t)$. The following states the detailed steps about our reconstruction approach.

**Algorithm 3:**

**Step1.** Give the sampling value *y*_*g*_(*t*) of the end-to-end network traffic.

**Step2.** Using Algorithm 1, obtain the fractal interpolation results ${\hat{y}}_{f}^{}$.

The article "Fine-granularity inference and estimations to network traffic for SDN" was retracted in 2025. Reasons: unreliable results or conclusions; concerns about the peer review; concerns about the article.

**Step3.** According to Algorithm 2, get the cubic spline interpolation result ${\hat{y}}_{c}^{}$.

**Step4.** Using Eq (24), determine the optimal weighted coefficient *b* and build the weighted geometric average model shown in Eq (19).

**Step5.** For the new sampling value *y*_*g*,*new*_(*t*), attain the accurate reconstruction result $\hat{y}(t)$ of the end-to-end network traffic according to Eq (19).

In short, we have proposed three algorithms to obtain the fine-granularity accurate end-to-end traffic reconstruction and estimation from the coarse-granularity sampled data. Algorithm 1 is used to establish the fractal interpolation reconstruction and estimation, while algorithm 3 are utilized to attain the cubic spline interpolation result. Based on Algorithms 1–2, Algorithm 3 is exploited to reconstruct the total resulting estimation.

## Simulation results and analysis

To verify our reconstruction approach to the end-to-end network traffic for SDN applications, simulation experiments use the real data from the Abilene network [13] that contains 12 nodes and 144 end-to-end flows. We use the Mininet simulation platform to simulate the SDN application. In our simulation, we simulate the Abilene network topology and take the real data from it as the input of our simulation topology. The TomoGravity [14], PCA [22] and SRSVD [1] methods are reported as accurate methods for the reconstruction of end-to-end traffic. Here, we compare the proposed fractal interpolation reconstruction method proposed (Algorithm 1), the proposed cubic spline interpolation reconstruction method (Algorithm 2), and the proposed weighted geometric average reconstruction method (Algorithm 1). Then, we also analyze the reconstruction errors, including the spatial relative errors (SREs), the temporal relative errors (TREs), and the cumulative distribution function (CDF) of the SREs and TREs. Concurrently, we analyze the impact of the different sampling granularities on the reconstruction performance and discuss the performance improvement of our three methods compared to previous methods.

### Reconstruction of network traffic

Figs 3, 4 and 5 respectively denote the reconstruction results of the Origin-Destination (OD) (or end-to-end) flows when the time sampling granularity is 1 hour, 4 hours, and 8 hours. We reconstruct the network traffic for every five minutes within seven days. For different sampling granularities, we draw two OD flows. Each OD flow shows a comparison of the reconstructed value and the true value. The figures show the reconstructed value obtained by the three methods proposed in this paper and the three methods mentioned in the literature, where the Pink line indicates the real value. The Fractal, Spline and Geometry methods are represented by the dark green, ink blue and bright blue lines, respectively. The SRSVD, TomoG, and PCA methods are indicated with blue, yellow and green lines, respectively. Comparing the differences between the true value and the reconstructed value shown in each figure, we have come to the following three conclusions. First, Figs 3, 4 and 5 show that the reconstructed value of the Fractal, Spline and Geometry methods are closer to the true value, and their reconstruction results are superior to those of the SRSVD, TomoG and PCA methods. Second, by comparing Fig 3A, Fig 4A and Fig 5A, we see that with the increase of sampling granularity (from 60 minutes to 8 hours), the reconstruction results of the Fractal Method slightly worsen, but they are still better than those of the SRSVD, TomoG and PCA methods. Comparing subfigures (b) and (c) in Figs 3, 4 and 5, the Spline and Geometry methods reach the same conclusion. Third, from Figs 3, 4 and 5, we find that the geometry method is superior to the Fractal and Spline methods and much closer to the true value of the end-to-end network traffic.

The article "Fine-granularity inference and estimations to network traffic for SDN" was retracted in 2025. Reasons: unreliable results or conclusions; concerns about the peer review; concerns about the article.

**Fig 3:** Reconstruction results of end-to-end network traffic from the 60-minute time granularity to 5-minute.

**Fig 4:** Reconstruction results of the end-to-end network traffic from the 4-hour time granularity to 5-minute.

**Fig 5:** Reconstruction results of the end-to-end network traffic from the 8-hour time granularity to 5-minute.

### Reconstruction error analysis

In the reconstruction of the end-to-end traffic, the SREs indicate the spatial relationships between the reconstruction error and the end-to-end flow and reflects the reconstruction accuracy of the reconstruction method in space. The TREs show the change in the reconstruction error over time and reflects the reconstruction accuracy of the reconstruction method in time. The SREs and TREs of the end-to-end traffic are important indicators to measure the reconstruction method. They are defined as follows:

$$\left\{ \begin{array}{c} err_{sp}(n)=\frac{||{\hat{x}}_{N}(n)-x_{N}(n)|{|}_{2}}{||x_{N}(n)|{|}_{2}},\;n=1,2,\ldots ,u\\ err_{tm}(t)=\frac{||{\hat{x}}_{u}(t)-x_{u}(t)|{|}_{2}}{||x_{u}(t)|{|}_{2}},\;t=1,2,\ldots ,N \end{array}\right.$$ (27)

where *err*_*sp*_(*n*) and *err*_*tm*_(*t*) denote the SRE and TRE for node pairs *n* and at time slot *t*, respectively; *u* and *N* represent the node pairs' and measurement time slots' number.

Figs 6, 7 and 8 show the SREs and TREs of the end-to-end network traffic reconstruction using the Fractal, Spline, Geometry, SRSVD, TomoG, and PCA methods from the 60-minute, 4-hour, and 8-hour time granularities to the 5-minute one. From Fig 6A, 6B and 6C, we see that for the network traffic reconstruction from the 60-minute to the 5-minute time granularity, our proposed three methods have lower SREs and TREs than the SRSVD, TomoG, and PCA. Moreover, in contrast to the SRSVD, TomoG, and PCA, the SREs of our three methods are lower and have no large fluctuations. This indicates that our three methods can perform more accurate and robust reconstructions of the end-to-end network traffic from 60 minutes to 5 minutes for all end-to-end flows than the SRSVD, TomoG, and PCA. Similarly, the TREs of our three methods are lower and also have no large fluctuations. This also indicates that our three methods can perform more accurate and robust reconstructions of the end-to-end network traffic from 60 minutes to 5 minutes for all reconstruction time slots than the SRSVD, TomoG, and PCA. More importantly, the SREs and TREs of the fractal, spline and geometry methods are all respectively below 0.4 and 0.15. In our three methods, Fig 6D illustrates that the SREs and TREs of the geometry method are the lowest, but those of the fractal and spline methods are nearly identical. This is consistent with our expectations. Thus, for the reconstruction of the end-to-end network traffic from the 60-minute to the 5-minute, our three methods hold lower reconstruction errors.

The article "Fine-granularity inference and estimations to network traffic for SDN" was retracted in 2025. Reasons: unreliable results or conclusions; concerns about the peer review; concerns about the article.

**Fig 6:** The SREs and TREs of the six methods from the 60-minute time granularity to the 5-minute one.

**Fig 7:** The SREs and TREs of the six methods from the 4-hour time granularity to the 5-minute one.

**Fig 8:** SREs and TREs of six methods from 8-hour time granularity to 5-minute one.

From Fig 7A, 7B and 7C, we see that for the network traffic reconstruction from the 4-hour to the 5-minute time granularity, our proposed three methods hold lower SREs and TREs than the SRSVD, TomoG, and PCA. Moreover, compared with the SRSVD, TomoG, and PCA, the SREs of our three methods are lower and have no large fluctuations. This indicates that our three methods can perform more accurate and robust reconstructions of the end-to-end network traffic from 4 hours to 5 minutes for all end-to-end flows than the SRSVD, TomoG, and PCA. Similarly, the TREs of our three methods are lower and have no large fluctuations. This also indicates that our three methods can perform more accurate and robust reconstructions of the end-to-end network traffic from 4 hours to 5 minutes for all reconstruction time slots than the SRSVD, TomoG, and PCA. More importantly, the SREs and TREs of the fractal, spline and geometry methods are all respectively below 0.5 and 0.2. In our three methods, Fig 7D illustrates that the SREs and TREs of the geometry method are the lowest, but those of the fractal and spline methods are nearly identical. This is consistent with our expectations. Thus, for the reconstruction of end-to-end network traffic from 4 hours to 5 minutes, our three methods hold lower reconstruction errors.

The article "Fine-granularity inference and estimations to network traffic for SDN" was retracted in 2025. Reasons: unreliable results or conclusions; concerns about the peer review; concerns about the article.

From Fig 8A, 8B and 8C, we also see that for the network traffic reconstruction from the 8-hour to the 5-minute time granularity, our proposed three methods also hold lower SREs and TREs than the SRSVD, TomoG, and PCA. Moreover, in contrast to the SRSVD, TomoG, and PCA, the SREs of our three methods are lower and have no large changes. This shows that our three methods can make more accurate and robust reconstructions of the end-to-end network traffic from 8 hours to 5 minutes for all end-to-end flows than the SRSVD, TomoG, and PCA. Similarly, the TREs of our three methods are lower and also have no large fluctuations. This also suggests that our three methods can perform more accurate and robust reconstructions of the end-to-end network traffic from 8 hours to 5 minutes for all reconstruction time slots than the SRSVD, TomoG, and PCA. More importantly, the SREs and TREs of fractal, the spline and geometry methods are all respectively below 0.5 and 0.2. In our three methods, Fig 8D tells us that the SREs and TREs of the geometry method are lowest, but those of the fractal and spline methods are nearly identical. This is consistent with our expectations. Thus, for the reconstruction of end-to-end network traffic from the 8-hour to the 5-minute, our three methods hold lower reconstruction errors.

Figs 6, 7 and 8 show that for different time granularities of end-to-end network traffic, the curves of the SREs and TREs of our methods are all below those of the SRSVD, TomoG, and PCA. Moreover, the curves of the SREs and TREs of the geometry method are below those of the fractal and spline methods, but those of the fractal and spline methods are nearly overlapping. This indicates that our methods can perform more accurate reconstructions of the end-to-end network traffic, and the geometry method proposed in this paper exhibits the lowest construction error for all end-to-end flows and time slots.

### Impact of sampling granularity on performance

To more accurately evaluate the reconstruction results of these methods, here we discuss the impact of the sampling granularity on reconstruction performance by analyzing the CDFs of the SREs and TREs of these methods, namely, the CSRE (the CDFs of the SREs) and the CTRE (the CDFs of the TREs). Figs 9, 10 and 11 respectively denote the CSRE and CTRE of each method, with the sampling granularities of 60 minutes, 4 hours, and 8 hours. From Fig 9, for the 60-minute sampling granularity, we see that for the geometry, fractal, spline, TomoG, SRSVD, and PCA methods, the SREs of approximately 91%, 88%, 87%, 60%, 45%, and 42% of the end-to-end flows are below 0.5. Moreover, the TREs of approximately 80%, 67%, 58%, 0%, 0%, and 0% of the time slots are below 0.1. Furthermore, the curves of the CSRE and CTRE of the geometry, fractal, and spline methods are far above those of the TomoG, SRSVD, and PCA. That of geometry method is on the top. Similarly, from Fig 10, for the 4-hour sampling granularity, we see that for the geometry, fractal, spline, TomoG, SRSVD, and PCA methods, the SREs of approximately 82%, 81%, 80%, 60%, 45%, and 42% of the end-to-end flows are below 0.5. Moreover, the TREs of approximately 48%, 38%, 21%, 0%, 0%, and 0% of the time slots are below 0.1. Furthermore, the curves of the CSRE and CTRE of the geometry, fractal, and spline methods are far higher than those of the TomoG, SRSVD, and PCA. Moreover, that of the geometry method is on the top. From Fig 11, for the 8-hour sampling granularity, we see that for the geometry, fractal, spline, TomoG, SRSVD, and PCA methods, the SREs of approximately 80%, 79%, 75%, 60%, 45%, and 42% of the end-to-end flows are below 0.5. Moreover, the TREs of approximately 25%, 24%, 5%, 0%, 0%, and 0% of the time slots are below 0.1. The curves of the CSRE and CTRE of the geometry, fractal, and spline methods are far higher than those of the TomoG, SRSVD, and PCA. Again, that of the geometry method is on the top.

The article "Fine-granularity inference and estimations to network traffic for SDN" was retracted in 2025. Reasons: unreliable results or conclusions; concerns about the peer review; concerns about the article.

**Fig 9:** The CDF of the SREs and TREs with the 60-minute sampling granularity.

**Fig 10:** The CDF of the SREs and TREs with the 4-hour sampling granularity.

**Fig 11:** The CDF of the SREs and TREs with the 8-hour sampling granularity.

Figs 9, 10 and 11 show that as the sampling granularity of the end-to-end network traffic increases, the reconstruction errors of the geometry, fractal, and spline methods proposed in this paper also increase. This indicates that different sampling granularities can have impacts on the reconstruction performance for our methods, which is consistent with our expectations. Figs 9, 10 and 11 illustrate that, in contrast to the TomoG, SRSVD, and PCA, the geometry, fractal, and spline methods still possess more accurate reconstruction performance.

### Performance improvement

Figs 12, 13 and 14 illustrate the performance improvement ratios of the fractal, spline and geometry methods relative to the TomoG, PCA, and SRSVD when the sampling time granularities are 60 minutes, 4 hours, and 8 hours. From Fig 12, we discover that when the sampling time granularity is 60 minutes, the average performance improvement ratios of the fractal method to the TomoG, PCA, and SRSVD are up to 61.9%, 62.4%, and 65.5%, respectively. When the sampling time granularity is 4 hours, the average performance improvement ratios of the fractal method relative to the TomoG, PCA, and SRSVD are 53.7%, 54.3%, and 58.1%, respectively. When the sampling time granularity is 8 hours, the average performance improvement ratios of the fractal method relative to the TomoG, PCA, and SRSVD, are 43.9%, 44.6%, and 49.2%, respectively. This indicates that, in this scenario, the proposed fractal method holds the best reconstruction performance.

The article "Fine-granularity inference and estimations to network traffic for SDN" was retracted in 2025. Reasons: unreliable results or conclusions; concerns about the peer review; concerns about the article.

**Fig 12:** The performance improvement of the fractal relative to the TomoG, PCA, SRSVD.

**Fig 13:** The performance improvement of spline relative to the TomoG, PCA, SRSVD.

**Fig 14:** The performance improvement of the geometry relative to the TomoG, PCA, SRSVD.

Fig 13 illustrates that when the sampling time granularity is 60 minutes, the average performance improvement ratios of the spline method relative to the TomoG, PCA, and SRSVD are 64.7%, 65.8%, and 67.8%, respectively. When the sampling time granularity is 4 hours, the average performance improvement ratios of the spline method relative to the TomoG, PCA, and SRSVD are 57.9%, 59.2%, and 61.6%, respectively. When the sampling time granularity is 8 hours, the average performance improvement ratios of the spline method relative to the TomoG, PCA, and SRSVD are 54.1%, 55.6%, 58.2%, respectively. This suggests that, in this scenario, the proposed spline method exhibits the most accurate reconstruction performance.

From Fig 14, we can see that when the sampling time granularity is 60 minutes, the average performance improvement ratios of the geometry method relative to the TomoG, PCA, and SRSVD are 66.5%, 67.0%, and 69.7%, respectively. When the sampling time granularity is 4 hours, the average performance improvement ratios of the geometry method relative to the TomoG, PCA, and SRSVD are 58.9%, 59.5%, and 62.8%, respectively. When the sampling time granularity is 8 hours, the average performance improvement ratios of the geometry method relative to the TomoG, PCA, and SRSVD are 53.0%, 53.6%, and 57.4%, respectively. This suggests that, under this scenario, the proposed spline method has the best reconstruction performance.

## Conclusion

This paper studies how to recover the end-to-end network traffic in fine time granularity from the sampled traffic traces in high-speed backbone networks for SDN applications. By taking advantage of the fractal and self-similar features of the end-to-end network traffic, we use the fractal interpolation method to recover them in the finer time granularity. Concurrently, we also use the cubic spline interpolation method to reconstruct the end-to-end network traffic in the finer time granularity. To fully exploit the advantages of the two reconstruction methods proposed in this paper, we account for the weighted geometric average process to improve the reconstruction accuracy of the end-to-end network traffic. By combining both of the presented reconstruction methods, we propose the third reconstruction approach for the end-to-end network traffic. Simulation results show that our approaches hold the best reconstruction performance.
